# Towards Tough Thermoplastic Adhesive Tape by Microstructuring the Tape Using Tailored Defects

**DOI:** 10.3390/polym15020259

**Published:** 2023-01-04

**Authors:** Ahmed Wagih, Hassan A. Mahmoud, Ran Tao, Gilles Lubineau

**Affiliations:** 1 Mechanical Engineering Program, Physical Science and Engineering Division, King Abdullah University of Science and Technology (KAUST), Thuwal 23955-6900, Saudi Arabia; 2 Mechanics of Composites for Energy and Mobility Lab, King Abdullah University of Science and Technology (KAUST), Thuwal 23955-6900, Saudi Arabia

**Keywords:** thermoplastic adhesive tapes, adhesive joints, fracture toughness, damage mechanics, modeling

## Abstract

This paper presents a strategy towards achieving thermoplastic adhesive tapes with high toughness by microstructuring conventional tapes using tailored defects. Toughened tape was manufactured using two layers of a conventional tape where the bondline between the two adhesive layers was microstructured by embedding tailored defects with specific size and gap between them using PTFE film. Mode I toughness of the toughened tape was characterized experimentally. A high-fidelity finite element model was implemented to describe the toughening mechanisms using double cantilever beam simulations and end notch flexural tests. The model considers for the plasticity of the adhesive layer, the decohesion at the adherend–adhesive and adhesive–adhesive interfaces and progressive damage inside the adhesive layer. The adhesive–adhesive interface with the tailored defects inside the adhesive layer enables crack migration between adherend–adhesive interfaces, crack propagation at adhesive–adhesive interface, backward crack propagation under the defect, and plastic deformation of the adhesive ligament. The maximum toughness improvement of the tape with tailored defects of equal width and gap between two successive defects of 2 mm reached 278% and 147% for mode I and II, respectively, compared to conventional tape.

## 1. Introduction

Adhesive bonding is one of the most common techniques to assemble primary and secondary structures; and commonly applied in primary structures, such as aircraft wings, body panel stiffeners, automobile parts assemblies, etc. [1]. It is also used in modern civil engineering structures assembly and internal structures for many purposes [2,3], and widely used in medical applications, such as wound dressing, electrode-attachment for electrocardiogram tests, and transdermal drug delivery system [4]. Many adhesives classifications have been proposed depending on origin material (natural, synthetic), curing process (physical, chemical), usage (structural, non-structural), and matrix type (thermoset or thermoplastic), which has been the most common classification.

Thermoset adhesives are commonly employed for structural applications and usually cured using chemical or mixed chemical and physical processes. The bonding process includes adherends surface preparation, applying adhesive, bonding the adherends, applying pressure, and curing for relatively long periods. Once cured, the adherends can hardly be separated. This class of adhesives has received considerable attention due to wide applications for aerospace and aircraft structures [5], with many developments to improve the structural integrity and toughness for thermoset-based adhesive joints, including interleaving [6,7], fiber stitching [8,9], Z-pinning [10,11], and substrate treatment [12,13,14]. Our research group has previously made significant contributions in this regard, developing three distinct techniques to improve toughness and structural integrity for thermoset-based adhesive joints. The first technique is by modifying adherends microstructure using laser-based heterogeneous surface treatments. In this technique, we demonstrated that creating an alternating pattern of high- and low-power laser treatment on adherend surfaces improves mode I and II toughness (the most common failure modes) 3 and 2 fold, respectively, compared with untreated joints [15,16]. The improvement was due to activating non-local damage mechanisms that dissipate energy during loading, including generating secondary cracks, and adhesive ligament formation and breakage. Applying this technique to structural T-joint achieves 2- and 15-fold improvement in joint strength and toughness, respectively, compared with untreated T-joints [17]. The second technique is by toughening the thermoset adhesive bond line using thermoplastic carriers [18]. The employment of this technique for adhesive joints provides 3.5-fold improvement compared with the pure thermoset-adhesive joints due to the high plasticity of the thermoplastic carrier that dissipates more energy during deformation. The third method is mimicking biological adhesion systems in the adhesive bonding, such as gecko and mytiluscalifornianus, by introducing sacrificial cracks inside the bond line that mimic voids in biological adhesion systems [19,20]. This technique results in an improvement of the mode I and II toughness by 1.5- and 2-fold, respectively, compared with conventional joints. The employment of this technique to structural T-joint achieves 3.3- and 18.9-fold improvement in joint strength and toughness, respectively, compared with classical T-joints [21].

Thermoplastic adhesive tapes can also be used for fast bonding, where the joint does not require long curing time or specific curing conditions [22], making them ideal for construction and medical applications. For construction purposes, the tapes were used for sealing diffusion film joints between roof elements and concrete floors with masonry blocks; and ensuring building air-tightness at doors and windows, preventing air entering air-conditioned buildings, which has a major role in energy efficiency for state-of-the-art buildings [3,23,24]. For medical purposes, adhesive tapes were widely used for manufacturing human joint supports and wound dressings. Once the thermoplastic adhesive tape is placed between the adherends, the joint can sustain the maximum load without requiring curing, which is an advantage over thermoset-based adhesives. Most adhesive tapes are formed mainly from two components: adhesive and carrier or matrix. The choice between adhesives is very limited, with only three main types: rubber, acrylic, and silicon. Rubber adhesives are mainly used for low-stress requirements, such as indoor applications, whereas acrylic adhesives can be applied for higher stress requirements with long-term bonding. Silicon adhesive is the most expensive with very good adhesion and high-temperature resistance [25]. In contrast, many materials can act as a carrier for the adhesive, including PET, PE, PP, PVC, woollen cloth, etc. Most current techniques to improve thermoplastic adhesive tapes toughness change of the matrix material (carrier) that might allow plasticity of the joint during deformation [26]. However, this approach cannot be applied to medical tapes, where specific adhesives and matrices must be selected for contact with human skin. Specifically for joint supports, where, in some cases, the healing process last for month, while the adhesive joint support only last for a maximum of 3 days [4], which require frequent change on the injured joint and, thus, affect the healing process.

Therefore, this study considered toughening thermoplastic adhesive tapes without changing the matrix or adhesive material. The proposed method considers microstructuring the tape using tailored defects. Embedding defects between two adhesive layers allows local deformations between adhesive layers, and dispersing the damage at adherend–adhesive and adhesive–adhesive interfaces that enhances joint toughness. Mode I tape toughness was characterized using the double cantilever beam (DCB) test. DCB and end notch flexural (ENF) responses for conventional and toughened tapes were simulated using a high-fidelity finite element (FE) model that looks for damage inside the adhesive layers and at adhesive–adherend interfaces. We subsequently performed a parametric study using the developed model to optimize the tape microstructure.

## 2. Methods

### 2.1. Manufacturing Toughened Thermoplastic Adhesive Tape

Toughened thermoplastic tapes were manufactured using conventional 0.25 mm thick thermoplastic tapes (3M high-performance double coated tape 9087). Figure 1a shows the thermoplastic double tape comprised two adhesive layers over a carrier from both sides. To manufacture the toughened tapes, PTFE films (defect) were placed over each tape with certain gap between them as shown in Figure 1a. Figure 1b shows the proposed toughened tape included two subadhesive tapes, each comprising an adhesive layer over a carrier. The subadhesive tapes were placed over each other and defects were tailored in their interface between them. We employed an 18 μm thick PTFE film to generate defects. Thus, manufacturing the toughened tapes included four steps. In the first step, one cover was removed from the first conventional tape. Then, in the second step, PTFE film with designed width *c*, and gap between films *g*, was placed over the tape, see Figure 1a. Hence, the distance between two successive PTFE films over conventional tapes equals *g*. After placing this PTFE film, it was pressed over the conventional tape to generate kind of offset between defects on the adhesive bondline, see Figure 1a. This offset was generated based on our previous study on bioinspired thermoset adhesive, where the finite element simulations demonstrated the benefit from an offset between defects in improving mode I toughness [20]. For comparison, we manufactured a tape composed of two 3M thermoplastic adhesive tapes without embedding defects that is called conventional tape.

Adherends for characterizing mode I toughness were made from unidirectional carbon/epoxy (T700/M21 Hexply, Hexcel) prepregs. Eight 0.25 mm thick plies were stacked with the same orientation (0${}^{\circ }$) to obtain 2 mm thick adherends. The prepregs were cut into 300 × 300 mm${}^{2}$ squares and stacked using the hand lay-up technique over a peel-ply surface. Stacked plates were cured using compression molding at 7 bar and 180 ${}^{\circ }$C for 2 h with 3 ${}^{\circ }$C/min heating and cooling rates using a hydraulic hot press. After curing, the DCB samples of 150 × 20 mm${}^{2}$ were cut from the plates using a water jet machine. Finally, the DCB samples were cleaned using acetone to remove any contaminants and bonded as shown in Figure 1c,d.

### 2.2. Experimental Tests

To characterize mode I toughness for the toughened adhesive tapes, DCB tests were performed following the ASTM D5528-13 standard. Figure 2 shows the experimental test setup performed using a universal testing machine (Instron 2885) at 1 mm/min loading rate. Samples were loaded through aluminum blocks that were bonded to the adherends using Araldite A/B adhesive. A high-resolution camera captured real time crack propagation and damage modes during the testing. Four samples were tested for each batch and the average toughness was computed.

### 2.3. Finite Element Modeling of DCB and ENF Tests

DCB and ENF responses were simulated using a two-dimensional (2D) plane-strain FE model implemented on Abaqus standard, as shown in Figure 3. High-fidelity FE models that simulate both responses were generated considering the real volume and microstructure for the adhesive layer to predict the different damage modes inside the adhesive layer. This model superior to conventional modeling, where the adhesive layer is treated as a single layer of cohesive elements. Conventional models only considers intrinsic toughness of the interface, which can be valid in the case of thin layer adhesives with very low plasticity. However, conventional models are invalid for thermoplastic tapes with sacrificial defects, where high plasticity and allowable damage growth inside the adhesive layers exist. Therefore, the high-fidelity FE models consider intrinsic and extrinsic toughness for the adhesive interface to tackle these problems. The adhesive layer comprised two sub-layers to simulate the manufactured tapes, where mechanical responses for each sub-layer were defined using an elastic-plastic model.

Figure 3 shows the elastic response extends until yield strength $\sigma_{y}$ is reached, then an isotropic strain hardening model applies until tensile strength $\sigma_{u}$ is attained. Damage grows following a linear softening when exerted stresses exceed adhesive ultimate strength until failure strain is attained. A vertical softening law is then defined to reach complete failure as shown in Figure 3c. Stress–strain responses for the thermoplastic adhesive tapes were obtained using a standard tensile test, and the following parameters were input to the model: *E* = 210 MPa, $\sigma_{y}$ = 6.00 MPa, ν = 0.325 and $\sigma_{u}$ = 12.59 MPa. Adherends were defined using an orthotropic linear elastic model with $E_{xx}$ = 125 GPa, $E_{yy}$ = 7.8 GPa, $G_{xy}$ = $G_{xz}$ = 5.1 GPa, $G_{yz}$ = 2.79 GPa, $\nu_{xy}$ = $\nu_{xz}$ = 0.33, and $\nu_{yz}$ = 0.4. These properties were extracted our previous work, which included full characterization [20]. Q4 plane strain elements (CPE4R) with reduced integration were used for meshing the adherends and adhesive.

The interaction between adhesive sub-layers and adherends was defined using bilinear cohesive elements as shown in Figure 3c. Damage initiation was governed by the maximum stress criterion. Cracks initiate at the interface when normal or shear stresses reach critical stress $\sigma_{c}$ and propagate following the mode independent criterion (mode I or mode II) depending on the applied stresses at the interface, with opening and shear fracture energy $G_{I}$ and $G_{II}$, respectively. Mode I fracture energy and critical stresses for the adhesive–adherend interface (cohesive elements #1 in Figure 3c) were characterized as $G_{I}$ = 0.018 N/mm and $\sigma_{cI}$ = 0.2 MPa (see Section 2.5 for details). Mode II fracture energy was considered twice compared with mode I toughness, and critical stress was computed using the analytical expression derived elsewhere [27,28] and equals 1.38 MPa. Cohesive parameters for the interface between the two sub-adhesive layers (cohesive elements #2 in Figure 3) were characterized as $G_{I}$ = 0.045 N/mm and $\sigma_{cI}$ = 0.5 MPa in mode I with $G_{II}$ = 0.09 N/mm and $\sigma_{c}II$ = 2.18 MPa. Cohesive element stiffness was constant for both interfaces and obtained as the ratio between adhesive stiffness and cohesive element thickness, which equals 2.1 × 10${}^{6}$ Pa. The first cohesive element at the upper adhesive–adherend interface was defined with weak cohesive properties ($\sigma_{cI}$ = 0.05 MPa and *G* = 0.0001 N/mm) to ensure crack initiation at the upper interface. This mimics the experiments where a pre-crack was generated at that interface.

Sacrificial defects were defined using cohesive elements with weak cohesive properties as well. Defects were defined at the peaks of the waves, to achieve 10 μm offset between successive cracks, as previously suggested by the authors [20]. Mesh sensitivity was studied by employing four element widths at the interface: 50, 100, 150, and 200 μm, resulting in models with 51,902, 26,492, 18,029, and 13,787 elements. The models were solved using a standard implicit solver. A 7 mm opening was prescribed to the left end of the DCB beam, while the x-displacement was fixed at zero. For ENF test simulation, a displacement in z-direction of 2 mm was applied to a pilot node attached to the rigid indenter, while the x-displacement was fixed at zero.

Parametric studies using these models investigated effects from defect width and gap between two successive cracks on mode I and II toughness. Defect width effect was investigated for fixed gap equals 5 mm, while defect width equals 1, 2, 3, 4, and 5 mm. Gap size effect on toughness was investigated with fixed defect width equals 2 mm, while gap width equals 1, 2, 3, 4, and 5 mm.

### 2.4. Data Reduction Methods for Mode I and II Fracture Toughness

Mode I and II R-curves were computed based on the simple beam theory using the load-displacement response from DCB and ENF tests, respectively. We used an effective crack length-based data-reduction method to overcome difficulties monitoring crack growth during loading. This method does not require any experimental information on the crack growth. Mode I R-curve was constructed using the Hashemi et al. [29] solution with fracture toughness $G_{I}$ and effective crack length $a_{I}$ expressed as:

(1) $$G_{I}={\left[\frac{9}{4}\frac{P^{4}\cdot \delta^{2}}{B^{3}\cdot E_{xx}\cdot I}\right]}^{\frac{1}{3}}$$

(2) $$a_{I}={\left[\frac{\delta \cdot B\cdot h^{3}\cdot E_{xx}}{8P}\right]}^{\frac{1}{3}}-\zeta \cdot h$$

where *P* is the load, δ is the applied displacement at loading point; *B* is the sample width; $E_{xx}$ is the in-plane modulus in the fiber direction; *I* is the second moment of area; *h* is the adherend thickness; and ζ is a correction factor that compensates for the assumption that compliance at the crack root is zero, which differs from the real response where some deflection and rotation occur at the crack tip [30,31].

Thus, ζ can be computed as:

(3) $$\zeta ={\left(\frac{E_{xx}}{11G_{xy}}\right)}^{\frac{1}{2}}{\left[3-2{\left(\frac{\gamma }{1+\gamma }\right)}^{2}\right]}^{\frac{1}{2}}$$

where $\gamma =\frac{1.18}{G_{xy}}{\left(E_{xx}\cdot E_{yy}\right)}^{\frac{1}{2}}$, $E_{yy}$ is the in-plane modulus in the direction perpendicular to fiber direction and $G_{xy}$ is the in-plane shear modulus.

For mode II R-curve, specimen compliance *C* can be expressed as [32]:

(4) $$C=\frac{\delta }{P}=\frac{3a_{II}^{3}+2L^{3}}{8Bh^{3}E_{xx}}$$

and effective crack length $a_{II}$ as:

(5) $$a_{II}={\left[\frac{8\delta Bh^{3}E_{xx}}{3P}-\frac{2}{3}L^{3}\right]}^{\frac{1}{3}}$$

Then, from linear elastic fracture mechanics, $G_{II}=\frac{P^{2}}{2B}\frac{dC}{da}$, and hence mode II fracture toughness can be expressed as:

(6) $$G_{II}=\frac{9P^{2}a_{II}^{2}}{16B^{2}h^{3}E_{xx}}$$

### 2.5. Characterizing Cohesive Laws for Interfaces

In order to fully define the cohesive elements properties, fracture toughness $G_{I1}$ and interfacial strength $\sigma_{cI1}$ should be measured for the interface. Fracture toughness for cohesive elements #1 was determined experimentally using DCB tests, where the bonding procedure from Section 2.1 was applied to bond the DCB samples. In these samples, cracks propagated only at the adherend–adhesive interface. Measured load-displacement data were used to predict the R-curve using the data reduction method from Section 2.4. Thus, calculated mode I toughness was $G_{I1}$ = 0.018 N/mm.

To determine the interfacial strength, we run the developed FE model with different values of $\sigma_{cI1}$ until achieving best fitting with experimental results as shown in Figure 4. Best fit interfacial strength was $\sigma_{cI1}$ = 0.2 MPa. To characterize the cohesive properties of the cohesive elements #2, we glued thermoplastic tapes to adherends using Araldite 420 A/B adhesive, which has higher toughness than the thermoplastic tape. We then bonded the adherends already pre-equipped with thermoplastic tapes to ensure crack prorogation at the interface between the two adhesive sublayers (interface #2). Thus, the calculated toughness was $G_{I2}$ = 0.045 N/mm. We followed the same procedure as for $\sigma_{cI1}$ to obtain optimized interfacial strength for this interface $\sigma_{cI2}$ = 0.5 MPa.

## 3. Results

Figure 5 shows mesh sensitivity analysis for DCB test simulations considering four different mesh sizes. Differences between FE model predictions for the four meshes is very small. However, the model with largest mesh size exhibited slightly larger maximum load and lower displacement, whereas meshes with 0.1 and 0.05 mm element sizes showed an identical response. Thus, the adopted element size equal 0.1 mm for the parametric studies.

Figure 6 shows a comparison between the model prediction and DCB test results for conventional and toughened tapes with a 2 mm defect size and a 5 mm gap between defects. Figure 6a,b confirm fair agreement between the proposed model predictions and experimental measurements for conventional tape. For conventional tape, the initiation toughness of S01 and S02 was slightly higher than the FE model predictions because during our experiments we did not create a pre-crack at any of the interfaces. So, the initiation of the crack requires quite large energy to localize the stresses at one of the interfaces and then crack initiate at this interface. However, in the FE model, we presented the first cohesive element at the upper interface with weak cohesive element properties to initiate the crack at this interface and to avoid convergence issues. After the crack initiates, it propagates until the critical fracture toughness $G_{Ic}$ = 0.018 N/mm is reached. For the toughened tape, the model showed qualitative agreement with the experimental results. Since the PTFE locations are not as precise as those in the numerical model, and the viscosity of the thermoplastic adhesive, it is difficult to achieve perfect agreement with the experimental responses. It is even unrealistic to obtain identical experimental curves due to those variations. In the experiments, crack migrates to the lower adhesive–adherend interface at the first defect; whereas in the FE model prediction, the crack propagates at the upper interface after the first defect and migrates to the lower adhesive–adherend interface at the second defect. This is because the offset for the first crack was at the upper interface in the simulation, which inhibited crack migration at that defect. However, the crack migrates to the lower adhesive–adherend interface at the second defect, which was observed experimentally. The difference in the damage modes results in improved toughness to around 0.028 N/mm compared with 0.018 N/mm for the conventional tapes. The FE model is to capture the major failure mechanism and to help to better design the strategy. Here in Figure 6e, the FE model successfully reproduced the fracture mechanism found in experimental tests, that is the bridging ligaments due to the PTFE defects. Two main points were marked in the R-curve of the toughened tape (see Figure 6d), $G_{IT}$ and $G_{Ic}$, which represent total energy in the system at this instant and the critical fracture energy, respectively. The difference between them is elastic energy stored in the system during propagation, associated with the presence of defects. Hence, treating both points should be done with caution for real structures, where $G_{IT}$ can not be considered critical fracture toughness for the system since toughness reduced to almost half once the crack passed this point. The reason for this reduction is explained further in Section 4.

Figure 7 shows the effect of defect size, *c*, and the gap between successive defects, *g*, on load-displacement and R-curve for DCB joints made with the proposed toughened thermoplastic tape. Toughened tapes exhibit several load and toughness drops in their load-displacement and the R-curves compared with conventional tapes, which indicates crack arrest/jump during propagation. DCB response for toughened tapes is influenced by both *c* and *g*. Although, crack length has insignificant effect on critical fracture toughness of the tape, it affects total energy stored in the tape. However, *g* has no significant effect on fracture toughness except slightly smaller toughness improvement is achieved for the largest gap, 5 mm.

Figure 8 shows the effect of defect and gap sizes on the mode II response of toughened thermoplastic adhesive tapes. Both parameters affect the mode II toughness, where increasing the defect size improved the mode II toughness up to a certain value after which the effect was stabilized at $G_{IIc}$ = 0.045 N/mm compared to $G_{IIc}$ = 0.03 N/mm for conventional tape. For the gap between two defects, mode II toughness is proportional to the gap size up to 2 mm, after which the toughness decreases and stabilizes at a certain value for any other gap size.

## 4. Discussion

This section discusses different toughening mechanisms to clarify the observed responses of toughened thermoplastic adhesive tapes.

### 4.1. Toughening Mechanisms

Figure 9 shows toughening mechanisms for thermoplastic adhesive tape with *c* = 2 mm and *g* = 5 mm under DCB simulation. The figure shows the load-displacement curves for conventional and toughened tapes and the simulated crack growth at different stages of loading. Conventional tape exhibits typical crack propagation for DCB test, where the crack initiated at the upper adhesive–adherend interface and propagated along the same interface. In this case, load-displacement response is characterized by elastic load increase until the energy release rate exceeds the interface critical fracture toughness, then a crack initiates at the upper adhesive–adherend interface corresponding to point “1C” in Figure 9a. When this crack initiated, the load decreased while the crack propagates at the same interface as shown in Figure 9b, which is a typical response of DCB joints [20,28].

For the toughened tape, the response differs from the conventional tape. The crack initiates at the upper adhesive–adherend interface that corresponds to point “1T” in Figure 9a. Then the crack propagates until it reaches the first defect, where the main crack path is arrested, then the crack jumps over the defect, and a new crack is initiated in the same interface just after the defect. This crack jump causes the formation of an adhesive ligament that allows the crack to propagate along the adhesive–adhesive interface, increasing load up to “2T”. Initiating the new crack after the first defect dissipates more energy than propagating the already initiated crack. Hence, the crack at the upper interface propagates backward over the defect until reaches the end of the defect causing a sudden load drop in load-displacement response.

Thus, two main energy dissipation mechanisms occurred: new crack initiation after crack jump, and propagation of crack along the adhesive–adhesive interface. Some exerted energy was also stored in the system as elastic energy due to elastic deformation of the adhesive. This energy was released once the crack passed the defect, which causes a load drop in load-displacement response. If the elastic energy stored in the adhesive was the main cause for the increase in load and toughness up to point “2T”, the load would reduce back to the original response of conventional tape. However, this does not happen due to the aforementioned two dissipation mechanisms and the initiation of a crack at the lower interface which forms an adhesive ligament that initiate storing of elastic energy again. The restoration of the elastic energy at the first defect resulted in initiation of a crack at the lower adhesive–adherend interface, as shown in Figure 9(c-3T); then load increased again with increasing displacement, while the crack propagated along the lower adhesive–adherend interface, forming a new adhesive ligament at the second defect (Figure 9(c-4T)). Formation of this ligament between the upper and lower adherends allows the main crack to propagate along the upper adhesive–adherend interface, and initiates a backward crack at the lower adhesive–adherend interface. The load increases with increasing the displacement due to dissipating the energy through growth of these cracks and the crack propagation along the adhesive–adhesive interface. Further increasing of the displacement, the crack migrates to the upper adhesive–adherend interface, again forming a new ligament with the same scenario: backward crack propagation and crack at the adhesive–adhesive interface until point “6T”. After this point, another load drop then occurs due to complete crack propagation over the second defect releasing part of the elastic energy stored inside the adhesive ligament. These damage modes for the conventional and the toughened tape were captured experimentally as well as shown in Figure 10.

Figure 11 shows toughening mechanisms in thermoplastic adhesive tape with *c* = 2 mm and *g* = 5 mm between successive defects under ENF testing. The adherends were removed from the model and the model was extruded to 20 mm wide for better readability of crack evolution. For conventional tape, crack initiates and propagates along the upper adhesive–adherend interface resulting reduction in the load as shown in Figure 11b. However, for the toughened tape, the evolution of crack propagation was different. The crack initiates at the upper adhesive–adherend interface and propagates until it reaches first defect, where the crack is arrested and the exerted energy stored as elastic deformation at the crack. The crack then jumps over the defect and starts propagating along the upper adhesive–adherend interface as shown in Figure 11(c-2T). Moreover, a new crack initiates at the lower adhesive–adherend interface after the defect. The initiation of new crack after the defect requires more fracture energy to initiate than propagation of an already initiated crack, leading to the load-displacement plateau response between points “1T” and “2T”. The cracks in the upper and lower adhesive–adherend interface propagate simultaneously, dissipating more energy until they reach the second defect. The same scenario that occurs as at the first crack, causing a crack jump, and increase in the applied displacement initiates another crack along the adhesive–adhesive interface as shown in Figure 11(c-4T), increasing energy dissipation as well. Thus, three toughening mechanisms contribute to toughening the tape.

The existence of defects in the toughened thermoplastic tape activate new energy dissipation mechanisms that enhance mode I and II toughness for the joint. Toughening mechanisms in mode I include the propagation of a crack at the adhesive–adhesive interface, backward crack propagation under the defect, and plastic deformation of the adhesive ligament. Toughening mechanism in mode II include crack jump and initiation of new crack after the defect, propagation of cracks at the upper and lower interfaces simultaneously, and propagation of crack along adhesive–adhesive interface.

### 4.2. Toughened Tape Microstructure Effects on Toughness

Figure 12 shows the effect of toughened thermoplastic adhesive microstructure on mode I and II toughness based on FE simulations, where $\bar{G}$ represents normalized toughness for toughened tape with respect to conventional tape. Both *c* and *g* influence mode I and II toughness improvement. Increasing *c* improves mode I and II toughness up to a certain limit. For the tape with *g* = 5 mm, the maximum mode I and II toughness improvement was achieved for *c* = 3 mm, where the mode I and II toughness improvement equal 227% and 160% conventional tape toughness, respectively. Further increasing *c* reduced the improvement of mode I toughness and stabilized the improvement rate in mode II toughness. Considering the toughening modes presented in Section 4.1, where the main crack propagates at the upper skin–adhesive interface, a backward crack propagates at the lower skin–adhesive interface, and a crack at the adhesive–adhesive interface, the relation between toughness increase and the crack length can be explained. Increasing *c* up to 3 mm, the backward crack propagation increases, while the length available for the adhesive–adhesive crack decreases. Despite this decrease in the propagation length at the adhesive–adhesive crack, the backward crack prorogation is larger, which globally enhances the toughness. Further increasing *c* more than 3 mm, the toughness reduction due to the reduction in the length available for the adhesive–adhesive crack became more significant which results in global toughness reduction. However, the toughness still is larger than the toughness of the baseline tape. For the tape with *c* = 2 mm, the maximum mode I and II toughness improvement was achieved for *g* = 2 mm, where the mode I and II toughness toughness equal 278% and 147% conventional tape toughness.

From the industrial point of view, the proposed toughened tapes is viable because it can be produced following the same manufacturing process as conventional tape, just adding an extra step of embedding PTFE film between the two adhesive layers. The proposed toughening strategy is also economically efficient since our simulations showed more than double toughness improvement by doubling the amount of adhesive matrix using a defect of *c* = 3 mm for a *g* = 5 mm and/or a defect *c* = 2 mm for a *g* = 2 mm, while for an experimental set, the improvement reaches 55%. The proposed concept can be applied for conventional tapes by embedding tailored defects between the adhesive and the matrix, which could also activate non-local damage mechanisms and hence toughness improvement with the same cost of the conventional tapes.

## 5. Conclusions

This paper presented a toughening strategy for thermoplastic adhesive tapes without changing any of the materials used for manufacturing conventional tape. The proposed strategy placed two layers of the same adhesive tapes over each other and embedding tailored defects with specific sizes and gaps between them at the bondline between the two adhesive layers. We used 3M high-performance double-coated tape to manufacture the toughened tapes, with PTFE film to generate defects at the adhesive–adhesive interface. A high-fidelity FE model was developed to simulate DCB and ENF responses. The developed model was validated experimentally, and simulated and measured results were employed to describe the toughening modes in detail. Toughened tape microstructure effects on mode I and II toughness were investigated by simulation using the developed FE model.

The proposed toughened tape exhibited greatly improved mode I toughness due to migration of crack between the two adhesive–adherend interfaces, propagation of crack at the adhesive–adhesive interface, backward crack propagation under the defect, and plastic deformation of the adhesive ligament. Toughening mechanisms in mode II include crack jump and initiation of new crack after the defect, propagation of cracks along the upper and lower interfaces simultaneously, and propagation of crack along adhesive–adhesive interface. Toughened tape microstructure highly influences toughness improvement rates, increasing mode I and II toughness with increased defect size and gap between successive defects up to a certain limit, then reducing to a plateau.

## Figures and Tables

**Figure 1:** Manufacturing toughened thermoplastic tapes and bonding DCB samples.

**Figure 2:** Experimental double cantilever beam test set up.

**Figure 3:** Two-dimensional models: (**a**) double cantilever beam (DCB), (**b**) end notch flexural (ENF) tests for bonded joints with thermoplastic adhesive tapes incorporating tailored defects, and (**c**) the cohesive interfaces and tailored defect details with tape’s stress–strain response.

**Figure 4:** Determining interfacial strength for cohesive elements #1.

**Figure 5:** Mesh sensitivity analysis for double cantilever beam (DCB) tests on toughened thermoplastic adhesive tape with 2 mm sacrificial defect and 5 mm gap: (**a**) load-displacement (P-δ) response; (**b**) fracture toughness, $G_{I}$-crack length, $a_{I}$ response (R-curve); and (**c**) meshes with different element sizes. the red lines in c represent the defects.

**Figure 6:** Proposed model prediction and experimental results for double cantilever bean test on: (**a**,**b**) conventional tapes, (**c**,**d**) toughened tape with 2 mm sacrificial defect and 5 mm gap, and (**e**) corresponding damage mode at 3 mm displacement for the toughened tape. In (**e**) the red lines represents the defect position and the blue arrows represent the crack propagation path.

**Figure 7:** Double cantilever beam (DCB) simulation crack width, *c* and gap between two successive cracks, *g* effects on, (**a**,**c**) load-displacement; and (**b**,**d**) R-curve, respectively.

**Figure 8:** End notch flexural (ENF) simulation crack width, *c*, and gap between two successive cracks, *g*, effects on, (**a**,**c**) load-displacement; and (**b**,**d**) R-curve, respectively.

**Figure 9:** Toughening mechanisms in thermoplastic adhesive tapes with 2 mm crack length and 5 mm gap between cracks: (**a**) load-displacement curves for double cantilever beam (DCB) simulation; and crack propagation in (**b**) conventional tape and (**c**) toughened tape.

**Figure 10:** Experimental evolution of toughening mechanisms in thermoplastic adhesive tapes with 2 mm crack length and 5 mm gap between cracks: (**a**) load-displacement curves for DCB test; and crack propagation in (**b**) conventional tape, and (**c**) toughened tape.

**Figure 11:** Toughening mechanisms in thermoplastic adhesive tapes with 2 mm defect length and 5 mm gap between defects: (**a**) load-displacement curves for end notch flexural (ENF) simulation; and crack propagation in (**b**) conventional, and (**c**) toughened tape.

**Figure 12:** Toughened thermoplastic adhesive tapes microstructure effects on mode I and II toughness with respect to the defect length *c* at a gap between successive defects *g* = 5 mm in (**a**) and *g* at *c* = 2 mm in (**b**). The analysis in the figure was extracted from the FE simulation.

## Data Availability

All the data will be available upon request.

## References

[1] Matthews F., Kilty P., Godwin E. (1982). A review of the strength of joints in fibre-reinforced plastics. Part 2. Adhesively bonded joints. Composites.

[2] Jucienė M., Dobilaitė V. (2021). Impact of climatic effects and various surfaces on the tack of adhesive tapes for building & construction. J. Build. Eng..

[3] Fufa S.M., Labonnote N., Frank S., Rüther P., Jelle B.P. (2018). Durability evaluation of adhesive tapes for building applications. Constr. Build. Mater..

[4] McNichol L., Lund C., Rosen T., Gray M. (2013). Medical adhesives and patient safety: State of the scienceconsensus statements for the assessment, prevention, and treatment of adhesive-related skin injuries. J. Wound Ostomy Cont. Nurs..

[5] Ageorges C., Ye L., Hou M. (2001). Advances in fusion bonding techniques for joining thermoplastic matrix composites: A review. Compos. Part A Appl. Sci. Manuf..

[6] Beckermann G.W., Pickering K.L. (2015). Mode I and Mode II interlaminar fracture toughness of composite laminates interleaved with electrospun nanofibre veils. Compos. Part A Appl. Sci. Manuf..

[7] Narducci F., Lee K.Y., Pinho S. (2018). Interface micro-texturing for interlaminar toughness tailoring: A film-casting technique. Compos. Sci. Technol..

[8] Jain L.K., Dransfield K.A., Mai Y.W. (1998). On the effects of stitching in CFRPs-II. Mode II delamination toughness. Compos. Sci. Technol..

[9] Mouritz A.P., Cox B. (2000). A mechanistic approach to the properties of stitched laminates. Compos. Part A Appl. Sci. Manuf..

[10] Chang P., Mouritz A., Cox B. (2006). Properties and failure mechanisms of pinned composite lap joints in monotonic and cyclic tension. Compos. Sci. Technol..

[11] Mouritz A.P. (2007). Review of z-pinned composite laminates. Compos. Part A Appl. Sci. Manuf..

[12] Fischer F., Kreling S., Jäschke P., Frauenhofer M., Kracht D., Dilger K. (2012). Laser surface pre-treatment of CFRP for adhesive bonding in consideration of the absorption behaviour. J. Adhes..

[13] Kanerva M., Saarela O. (2013). The peel ply surface treatment for adhesive bonding of composites: A review. Int. J. Adhes. Adhes..

[14] Leena K., Athira K., Bhuvaneswari S., Suraj S., Rao V.L. (2016). Effect of surface pre-treatment on surface characteristics and adhesive bond strength of aluminium alloy. Int. J. Adhes. Adhes..

[15] Tao R., Li X., Yudhanto A., Alfano M., Lubineau G. (2020). Laser-based interfacial patterning enables toughening of CFRP/epoxy joints through bridging of adhesive ligaments. Compos. Part A Appl. Sci. Manuf..

[16] Wagih A., Tao R., Yudhanto A., Lubineau G. (2020). Improving mode II fracture toughness of secondary bonded joints using laser patterning of adherends. Compos. Part A Appl. Sci. Manuf..

[17] Hashem M., Wagih A., Lubineau G. (2022). Laser-based pretreatment of composite T-joints for improved pull-off strength and toughness. Compos. Struct..

[18] Yudhanto A., Almulhim M., Kamal F., Tao R., Fatta L., Alfano M., Lubineau G. (2020). Enhancement of fracture toughness in secondary bonded CFRP using hybrid thermoplastic/thermoset bondline architecture. Compos. Sci. Technol..

[19] Wagih A., Lubineau G. (2021). Enhanced mode II fracture toughness of secondary bonded joints using tailored sacrificial cracks inside the adhesive. Compos. Sci. Technol..

[20] Wagih A., Tao R., Lubineau G. (2021). Bio-inspired adhesive joint with improved interlaminar fracture toughness. Compos. Part A Appl. Sci. Manuf..

[21] Wagih A., Hashem M., Lubineau G. (2022). Simultaneous strengthening and toughening of composite T-joints by microstructuring the adhesive bondline. Compos. Part A Appl. Sci. Manuf..

[22] Mapari S., Mestry S., Mhaske S. (2021). Developments in pressure-sensitive adhesives: A review. Polym. Bull..

[23] Langmans J., Desta T.Z., Alderweireldt L., Roels S. (2017). Durability of self-adhesive tapes for exterior air barrier applications: A laboratory investigation. Int. J. Vent..

[24] Jacobs V W.P., Daniel Dolan J., Dillard D.A., Ohanehi D.C. (2012). An evaluation of acrylic pressure sensitive adhesive tapes for bonding wood in building construction applications. J. Adhes. Sci. Technol..

[25] Schalau G., Bobenrieth A., Huber R.O., Nartker L.S., Thomas X. (2018). Silicone adhesives in medical applications. Applied Adhesive Bonding in Science and Technology.

[26] Petrie E.M. (2007). Handbook of Adhesives and Sealants.

[27] Song K., Dávila C.G., Rose C.A. Guidelines and parameter selection for the simulation of progressive delamination. Proceedings of the 2008 Abaqus User’s Conference.

[28] Turon A., Davila C.G., Camanho P.P., Costa J. (2007). An engineering solution for mesh size effects in the simulation of delamination using cohesive zone models. Eng. Fract. Mech..

[29] Hashemi S., Kinloch A.J., Williams J. (1990). The analysis of interlaminar fracture in uniaxial fibre-polymer composites. Proc. R. Soc. Lond. A Math. Phys. Sci..

[30] Kanninen M. (1974). A dynamic analysis of unstable crack propagation and arrest in the DCB test specimen. Int. J. Fract..

[31] Williams J. (1989). End corrections for orthotropic DCB specimens. Compos. Sci. Technol..

[32] Davies P., Sims G., Blackman B., Brunner A., Kageyama K., Hojo M., Tanaka K., Murri G., Rousseau C., Gieseke B. (1999). Comparison of test configurations for the determination of GIIc of unidirectional carbon/epoxy composites, an international round robin. Plast Rubber Compos..

